RETRACTED

# Migraine headache in Sudan

**DOI:** 10.1002/brb3.2429

**Published:** 2021-11-13

**Authors:** Etedal Ahmed A. Ibrahim, Ghada A. Mutaal Badri, Khabab Abbasher Hussien Mohamed Ahmed, Mohammed Eltahier Abdalla Omer

**Affiliations:** ^1^ Faculty of Medicine, Al Neelain University Department of Internal Medicine Khartoum Sudan; ^2^ The National Centre for Neurological Sciences Department of Neurology Khartoum Sudan; ^3^ Faculty of Medicine University of Khartoum Khartoum Sudan; ^4^ Faculty of Medicine and Health Sciences Department of Internal Medicine Gadarif University Gadarif Sudan

**Keywords:** aura, headache, migraine, precipitating factors, Sudan

## Abstract

**Background:**

Migraine is a main form of headache, it is also a chronic and complex neuroinflammatory disease; it is characterized by recurrent severe headaches, usually affecting one side of the head, and often accompanied by nausea and blurred vision. In susceptible individuals, irritants can trigger migraine attacks, which can be considered as triggers or accelerators.

**Objective:**

To describe the precipitating factors, clinical presentation, and treatment of migraine headache in Sudanese patients.

**Methods:**

This is a descriptive hospital‐based prospective study covering 130 patients during the study period from January 2016 to December 2018. At the National Centre for Neurological Science, Khartoum, participants were Sudanese patients with migraine headache after exclusion of other causes of headache. Data was collected using structured questionnaire entered and analyzed using SPSS version 22.0, p value < .05 is considered significant.

**Results:**

The study covered 130 study participants most of them were females (80%), within 26–35 years of age (56.9%) and a considerable proportion of them were housewives (40%). The majority of the study participants had headache without aura in 81.5% and headache with aura in 18.5% (mainly visual type 87.5%). Photophobia and nausea were the main associated symptoms in 51.5% and 50%, respectively. Acetaminophen was the main prescribed treatment in 46.1%, beta blockers was the main prophylaxis in 29.2%. Environmental triggers were the prevalent predisposing factors (43.8%) followed by fasting, lack of sleep, and exertion (24.6% for each).

**Conclusion:**

Environmental conditions were the commonest triggering factors of migraine headache, while Acetaminophen was the most common drug used for relieving migraine in this population.

## Abstract 2

This is a descriptive hospital‐based prospective study covering 130 patients during the study period from January 2016 to December 2018. At the National Centre for Neurological Science, Khartoum, participants were Sudanese patients with migraine headache after exclusion of other causes of headache.

RETRACTED

## 1 INTRODUCTION

Migraine is an intense and chronically repeated headache that is generally located to one side of the head, but can occur as a generalized throbbing headache with extension down to the neck or even the body. Clinically, there are different forms but migraine without aura (previously common migraine) is the commonest form. Migraine headaches can affect many people and women are slightly more susceptible than men. It is the second most common cause of headache, affecting approximately 15% of women and 6% of men (Macdonald, 2008).

It is featured by episodes of moderate to severe headache, which is often unilateral and pulsating and typically aggravated by routine physical activities. The timing of untreated migraine attacks is rather long, from 4 h to 3 days (median duration 18 h). Pain is accompanied by some other symptoms, the most common symptoms being nausea, vomiting, photophobia, and phonophobia. Other associated symptoms, such as osmophobia, pallor, fatigue, difficulty in concentration, blurred vision, or diarrhea may also be present (Norman, 2015).

There are numerous and varied potential headache precipitating factors (triggers). Not all triggers for migraine patients are stereotypes, and different seizures of the same person are not necessarily the same. Usually triggers can be from of a combination of many factors. For example, lack of sleep after a busy day at work or falling asleep the next morning can cause migraines. Other factors are thought to be alcohol and dehydration. The main groups of precipitating factors are: dietary (missing meals), stress, environmental (weather changes), hormonal (menses in women), head trauma, smoking, crying, sexual activity, smoke, smell, medications, sleep disturbances, as well as physical and emotional factors (Filho, 2002; Fragoso et al., 2003; Fukui et al., 2008; Holzhammer & Wöber, 2006; Macdonald, 2008; Spierings et al., 2001).

Although there is no clear evidence that certain dietary types my trigger migraine headache, some patients have reported some dietary elements like chocolate and cheese to lead to headache, but this can sometimes be part of food cravings and not the real cause of headache during the attack (Filho, 2002; Fragoso et al., 2003; Spierings et al., 2001).

Environmental triggers noticed include bright or flickering lights, bright sunlight, glare, overuse of computers, loud sounds, pollution, strong smells, for example, perfume, gasoline, chemicals, smoke‐filled rooms, various food odors, travel‐related stress, high altitude, flying, weather changes, and washing hair without subsequent good drying can also trigger intense migraine attacks (Macdonald, 2008; Robbins, 1994; Spierings et al., 2001; Zivadinov et al., 2003).

RETRACTED

The underlying mechanisms of migraine headache are not fully understood. It is, however, believed to contain the nerves and blood vessels of the brain. Initial recommended medication is with simple pain medication such as ibuprofen and paracetamol (Acetaminophen) for the headache, medication for the nausea, and the avoidance of triggers. Specific medications such as triptans or ergotamines may be used in the patients for whom simple pain medications are not functioning (Loder et al., 2013).

Therefore, in this study, we aimed to study precipitating factors, clinical presentation, and treatment of migraine headache in adult Sudanese patients.

## 2 METHODOLOGY

This study is a descriptive prospective hospital‐based study conducted at the National center for Neurological Science, Khartoum, Sudan, in the period from January 2016 to December 2018. The diagnosis of migraine headache was made based on the criteria of the International Headache Society for Migraine Headache (ICDH‐3). One‐hundred and thirty patients (aged more than 16 years) were enrolled in this study. Data was collected using questionnaire filled by the researcher and a physical examination check list.

### 2.1 Inclusion criteria

- Sudanese patients aged more than 16 years
- Patients with symptoms and signs of migraine headache according to international headache society for migraine headache
- **Without aura**
  A. At least five attacks fulfilling criteria B–D
  B. Headache attacks last from 4 to 72 h (without treatment or no treatment)
  C. Headache with at least two of the following four characteristics:
    1. Unilateral location
    2. Pulsating quality
    3. Moderate or severe pain intensity that inhibit or prohibits daily activities
    4. Symptoms are worsened by normal physical exertion such as climbing stairs
  D. In the case of a headache, at least one of the following symptoms occurs: Nausea, vomiting, photophobia, phonophobia cannot be better explained by other diagnoses ICHD‐3
- **With aura**
  A. At least two attacks that meet criteria B and C
  B. One or more of the subsequent completely reversible aura of mystery symptoms
    1. Visual
    2. Sensory
    3. Speech and or language
    4. Motor
    5. Brainstem
    6. Retinal
  C. At least two of the following four characteristics: At least one aura symptom spreads gradually within >5 min, and or two or more symptoms appear in sequence, each aura symptom lasts 5 to 60 min. At least one aura symptom and/or unilateral aura related symptoms or headache within 60 min immediately thereafter. Another diagnosis of ICHD does not better explain the headache. Transient ischemic attacks were excluded.

RETRACTED

Data was analyzed using statistical package for social sciences (SPSS) version (21.0) the results were represented in figures and graphs. The study was approved by the local ethical committee of the National Centre For Neurological Science. The patients were told that the information they received was anonymous and would only be used for this investigation. The consent of all participants were obtained.

## 3 RESULTS

A total of 130 migraine headache patients participated in the present study, 104 (80%) were females and 26 (20%) were males, the majority of them 74 (56.9%) found at the age group from 26 to 35 years and most of them 52 (40%) were housewives (Table 1). Most of the patients, 106 (81.5%), had migraine headache without aura and 24 (18.5%) had headache with aura (Table 2).

**TABLE 1:** Demographic characteristics distribution of the adult Sudanese patients with migraine headache (*n* = 130)

Demographic characteristics		Frequency	Percent
Age (years)	16–25	54	41.5
	26–35	74	56.9
	36–45	2	1.5
	>45	0	0
Sex	Male	26	20.0
	Female	104	80.0
Occupation	Housewife	52	40.0
	Worker	10	7.7
	Student	35	26.9
	Employee	32	24.6
	Out of work	1	0.8

**TABLE 2:** Clinical picture of the adult Sudanese patients with migraine headache

Clinical picture	Frequency	Percent
Headache with aura	24	18.5
Headache without aura	106	81.5
Total	130	100.0

Most of the aura was in visual type (87.5%), sensory (8.3%), and motor (4.2%) (Table 3).

**TABLE 3:** The distribution of the adult Sudanese patients with migraine headache according to their type of aura

Clinical picture	Frequency	Percent
Motor	1	4.2
Sensory	2	8.3
Visual	21	87.5
Speech	0	0.0
Total	24	100.0

Concerning the symptoms, the majority of the patients 59 (51.5%) had photophobia, 65 (50%) had nausea, 59 (45.4%) has phonophobia, and 56 (43.1%) had vomiting (Table 4).

**TABLE 4:** Symptoms' distribution among the adult Sudanese patients with migraine headache (*n* = 130)

Associated symptoms	Frequency	Percent
Nausea (yes)	65	50.0
Vomiting (yes)	56	43.1
Photophobia (yes)	67	51.5
Phonophobia (yes)	59	45.4

Acetaminophen was the main prescribed treatment in 60 (46.1%) patients, followed by Pizotifen combined with Acetaminophen in 56 (43.1%) patients and NSAID in only 14 (10.8%) patients (Table 5).

**TABLE 5:** The distribution of the adult Sudanese patients with migraine headache according to their treatment

Treatment	Frequency	Percent
Acetaminophen	60	46.1
NSAID	14	10.8
Pizotifen + Acetaminophen	56	43.1
Total	130	100

Beta blocker was the main prophylactic agents in 38 (29.2%) patients, antidepressant in 14 (10.8%) and antiepileptic in 3 (2.3%) patients (Figure 1).

RETRACTED

**FIGURE 1:** Distribution of prophylaxis among the adult Sudanese patients with migraine headache (*n* = 130)

In triggering factors, 43.8% of the patients had environmental triggers, 23.8% hormonal, 24.6% during fasting, 24.6% lack of sleep while 20% of them during stress and 15.4% of them dietary (Figure 2).

**FIGURE 2:** The distribution of the adult Sudanese patients with migraine headache according to triggers (*n* = 130)

As illustrated in Figure 3, more than half of the study participants (i.e., 71; 54.6%) had normal findings and the remaining 59 (54.6%) did not undergo imaging.

**FIGURE 3:** Imaging Findings of adult Sudanese patients with migraine headache depending on whether they received MRI imaging or not.

## 4 DISCUSSION

This is a cross‐sectional facility‐based study aimed to describe the precipitating factors, clinical presentation, and treatment of migraine headache. The study covered 130 study participants most of them were females (80%), more than half 56.9% were within 26–35 years of age, and a considerable proportion of them were housewives. Similar studies found that the migraine is common among the similar age group. (Ehsan, 2010) In Kurdish study, they realized that 33% of the patients were aged between 30 and 39 years, while 40.5% of patients experienced their first attack aged between 20 and 29 years.

Concerning the clinical presentation, the majority of the study participants had headache without aura in 81.5%, and most of the aura was in visual type 87.5%, with photophobia 51.5%, nausea 50%, and phonophobia in 45.4%. Other studies found (Stam et al., 2009) that nausea and vomiting usually occur later in the attack in about 80% and 50% of patients, respectively, along with anorexia and food intolerance. Some patients are pale and clammy, especially if they have nausea. Photophobia and/or photophobia are also associated with the headache. Lightheadedness is frequent.

Regarding the treatment, 61.1% of the study participants used Acetaminophen while 10.8% NSAIDs and 43.1% used Pizotifen + Acetaminophen. About 29.2% of them used B blockers as prophylaxis, 10.8% used anti‐depressants, and 2.3% used anti‐epileptic drugs. Other studies stated that (Ehsan, 2010) relief of migraine was achieved using NSAIDs in 50% of patients and sleep in 45.5%. Hence, 61% of the study population had positive family history of migraine, 32.5% of them reported maternal history of migraine. Other trials of non‐pharmacologic management have produced average reduction in migraines of 40%–50%, closely paralleling results obtained in trials of preventive drugs; however, the evidence base for non‐pharmacologic and pharmacologic prevention remains limited. A 16‐month randomized, placebo‐controlled trial by Holroyd et al. found that the combination of beta‐blocker therapy and behavioral management improved outcomes in patients with frequent migraines, while neither intervention was effective by itself (Le et al., 2011).

RETRACTED

The study participants had a variety of triggering factors. 43.8% had environmental triggers, 23.8% hormonal, 24.6% during fasting, 24.6% lack of sleep while 20% of them during stress. In the Kurdish study, they found that stress or psychological upset was the commonest triggering factor (80%), followed by increasing physical activity (68%), change in weather (65.5%), and in relation to fasting (65%) (Ehsan, 2010). Fasting in Ramadan was a triggering factor for headaches in 65% of patients. However, there was no significant association between the triggers of gender differences. Other studies found other factors such as lifestyle factors included alcohol consumption, smoking status, physical activity, and body mass index (Anke, 2011). Also, some researchers found (Wöber & Wöber‐Bingöl, 2010) that there is at least some evidence that environmental factors such as weather, lights, noise and odors, stress and other psychological factors, sleeping problems, fatigue and tiredness may play a role. In addition, drinking alcohol, quitting caffeine, skipping meals, and dehydration may cause migraines. This study found that more than half of the study participants had normal findings in imaging. As was known, computed tomography scanning of the head is indicated to rule out intracranial mass or hemorrhage in selected or atypical cases. A negative computed tomography scan may miss some small subarachnoid hemorrhages, tumors, and strokes, particularly those in the posterior fossa. A computed tomography scan without intravenous contrast also may miss some aneurysms. MRI and MRA are more sensitive for the detection of aneurysm or arteriovenous malformation that is not found in this study.

This study had some limitations. The relatively limited number of study participants (130 only) may negatively affect the probability of founding significant relationships between different factors and relevant circumstances and characteristics with the overall incidence of migraine among the risky patients.

Another limitation is follow‐up. Some outcomes may need to be followed over time for longer period. So, a long‐term cohort follow‐up design may be useful for more detailed description of the outcome.

## 5 CONCLUSION

This study concludes that females are predominately affected by migraine headache than males; the most affected age group ranged between 26 and 35 years. The most common presenting symptom was photophobia, and migraine headache was mainly presented without aura. Environmental conditions were the most frequent predisposing factor of headache in our study group. Moreover, the majority of patients received Acetaminophen as treatment and beta blockers as prophylaxis.

RETRACTED

### 5.1 Recommendations

Identifying triggers or predisposing factors is usually recommended as the main strategy for migraine management, and is considered an inexpensive way to reduce migraine.

## CONFLICT OF INTEREST

The authors declare no conflict of interest.

## AUTHOR CONTRIBUTIONS

All authors participated in planning the study, data collection, results, and discussion sections.

## FUNDING

This research did not receive any specific grant from funding agencies in the public, commercial, or not‐for‐profit sectors.

### PEER REVIEW

The peer review history for this article is available at https://publons.com/publon/10.1002/brb3.2429

## Data Availability

The materials datasets used and/or analyzed during this study are available from the corresponding author on reasonable request.
